# Assessment of C-Shaped Canal Morphology in Mandibular and Maxillary Second Molars in an Iraqi Subpopulation Using Cone-Beam Computed Tomography

**DOI:** 10.1155/2022/4886993

**Published:** 2022-03-16

**Authors:** Kazhan Abdalrahman, Ranjdar Talabani, Sara Kazzaz, Dlsoz Babarasul

**Affiliations:** Conservative Department, College of Dentistry, University of Sulaimani, Madam Mitterrand Street, Sulaimani, Iraq

## Abstract

Endodontic treatment is basically dependent on knowledge of the root canal anatomy. The goal of this study was to use cone-beam computed tomography (CBCT) imaging to examine the C-shaped canal configuration of mandibular and maxillary second molars in an Iraqi subpopulation. The prevalence and configurations of C-shaped canals were evaluated in 368 mandibular second molars and 369 maxillary second molars using CBCT scans. The effects of gender, age, and unilateral/bilateral on the presence of C-shaped canals were investigated. Chi-square and Fisher's exact tests were used to determine the level of significance (*p* ≤ 0.05), and kappa value was used to check reliability of results of the research. In mandibular second molars, the prevalence of C-shaped canals was 17.4%. The prevalence was significantly higher in females (23%) than males (10.4%) using the chi-square test. There is no significant difference in the prevalence of C-shaped canal depending on age and tooth position. The C2 type was the most common (56.3%). This prevalence did not differ with gender, age, or tooth position. In maxillary second molars, C-shaped canals were present in 7.9%. Type I (subtype C) (fusion of 2 root canals MB-DB) was the most common type of fused root (65.5%). There is no significant difference in the prevalence of C-shaped canal depending on the type of fused root, age, and tooth position. The majority of C-shaped canals in mandibular second molars were bilateral in both genders, but unilateral presence was more common in maxillary second molars in both genders. Within the limits of this study, C-shaped canals were found to be more common in mandibular second molars than in maxillary second molars in an Iraqi subpopulation.

## 1. Introduction

Root canal systems are complex anatomical structures that have significant consequences for root canal preparation. Various factors such as heredity and ethnic variances have been found to influence root canal morphology in the literature [1, 2]. Successful root canal therapy necessitates a thorough grasp of the morphology of the root canal system. For proper debridement, shaping, and complete obturation in three dimensions, knowledge of typical anatomy and variances from the norm is essential. The most common root canal shapes, as well as probable anatomic deviations, should be understood by clinicians [3]. The C-shaped canal configuration of the root canal system is one of the most challenging anatomical variances to comprehend. Because of its complex and unpredictable anatomy, particularly the form at the orifice level, the C-shaped canal poses a clinical challenge to endodontic operations in the middle and apical thirds of the root [4, 5]. It was first described using this term in 1979 by Cooke and Cox [6] and is named C-shaped because an axial plane of the canal resembles the letter “C,” and this system frequently exhibits webs, fins, and canal merging [7]. The failure of Hertwig's epithelial root sheath to fuse to the buccal or lingual root surface may be the primary cause of this anatomical anomaly, in which a continuous slit or web connects separate root canals [8]. The mandibular second molars have the most C-shaped canals, followed by the maxillary second molars, especially in Asian ethnic groups' dentition [9, 10].

In the literature, many methods for examining the root canal anatomy of the teeth have been published. For in vitro studies, the sectioning technique is the gold standard [11]. Other studies have shown that the cleaning method can be employed [12], while more recent studies have used microcomputed tomography [13]. Clinical results recorded under an operating microscope after access cavity preparation [14] or cone-beam computed tomography (CBCT) [15] are used in in vivo research. Because CBCT produces three-dimensional pictures that allow for a more accurate and detailed understanding of the root canal system than standard two-dimensional periapical radiography, cone-beam computed tomography (CBCT) has been proposed as a valuable approach for examining root canal architecture. The noninvasive nature of CBCT also allows for larger sample size study than previously allowed with microscopy research [16, 17].

This retrospective study investigated C-shaped canals found on CBCT in mandibular and maxillary second molars in an Iraqi subpopulation, with a focus on their prevalence, type, age, gender, and unilateral/bilateral occurrence.

## 2. Materials and Methods

### 2.1. Ethical Consideration

This study protocol was approved by the Ethics Committee of the University of Sulaimani College of Dentistry (No. 178).

### 2.2. Data Collection Procedure

The CBCT images of mandibular and maxillary second molars analyzed in this study were obtained from the database of the private B&R Dental Center, Sulaimani, Kurdistan Region/Iraq, for the period from February 2018 to May 2020. CBCT images from 368 mandibular second molars of 164 (44.6%) males and 204 (55.4%) females, with mean age 28.33 year old, and 369 maxillary second molars of 151 (40.9%) males and 218 (59.1%) females, with mean age of 32.86 year old, were assessed retrospectively, with age groups <30, 30-39, 40-49, and ≥50 years, all of which satisfied the following inclusion criteria:

1. Iraqi patients over 18 years old
2. Images containing mandibular and maxillary second molars with completely mature apex with no calcification
3. Images containing mandibular and maxillary second molars that had no caries, root filling, or postcrown restoration

### 2.3. Radiographic Examination

All CBCT images were acquired with a GALILEOS Sirona comfort PLUS unit (Sirona Dental Systems GmbH, Bensheim, Germany). Technical specifications were as follows: 15.4 cm spherical imaging volume, 0.25/0.125 mm isotropic voxel size, and a field of view of 15 cm diameter. The CBCT radiographs were taken according to the following parameters: 98 kVp, 3*e*5 mA, and exposure time of 14 s by Sidexis XG/Galileos implant software 1.9 (Dentsply Sirona). The CBCT images were examined using the built-in software package in an axial plane. If needed, image contrast and brightness were adjusted for optimal visualization. All the images were evaluated by two observers retrospectively.

The prevalence of C-shaped root canals according to age, gender, side, unilateral/bilateral occurrence, and correlation occurrence between mandibular and maxillary second molars was calculated.

The C-shaped canals was recorded when the floor of the pulp chamber floor could be seen. The canal shapes were classified as subtypes of C-shaped canal systems in mandibular second molars using Fan et al. modified Melton's technique as follows (Figure 1) [18]:

1. Category I (C1): the shape was an uninterrupted “C” with no separation or division
2. Category II (C2): the canal shape resembled a semicolon resulting from a discontinuation of the “C” outline, but either the *α* or *β* angle should be no less than 60° (Figure 2(a))
3. Category III (C3): two or 3 separate canals and both angles, *α* and *β*, were less than 60° (Figure 2(b))
4. Category IV (C4): a single round or oval canal
5. Category V (C5): no canal lumen could be observed

In maxillary second molars, the type of root fusion was classified by the sequence of root which was fused. The roots and canals were briefly referred with an abbreviation of capital letters, such as B, buccal root/canal; MB, mesiobuccal root/canal; DB, distobuccal root/canal; P, palatal root/canal; MP, mesiopalatal root/canal; and DP, distopalatal root/canal. The “-” between capital letters means fusion of roots or canals.

A total of 9 types of root fusion are described by Jo et al. [19] (Table 1). Therefore, this classification used in the present study started with dividing fusion of 2 roots and fusion of 3 roots. There were also some teeth with 2 or 4 roots, and those were classified into other types of root fusion. The difference between MB-DB-P and DB-MB-P was the sequence of fusion. The former made a C shape with the opening to the mesial side, but the latter made a C shape which opened to the distal side. Teeth that have palatal root fused with mesiobuccal and distobuccal roots were divided into 2 types. In MB-PDB (V shape) type, fusion was done in a serial manner and it looked like the letter “V.” In “all root” type, the cross-section image of the coronal portion looked like the letter “Y” or oval, and the cross-section image of the apical portion was circular.

### 2.4. The Standard Consistency Test (Kappa Value)

All samples were assessed for reliability testing by two observers, an endodontist and a radiologist, both of whom were highly skilled. A routine consistency check (kappa value) of the results was done at the same time.

When the kappa value was #0.4, reliability was considered unqualified; when the kappa value was between 0.41 and 0.6, reliability was considered moderate; when the kappa value was between 0.61 and 0.8, reliability was considered excellent; and when the kappa value was between 0.81 and 1.0, reliability was considered fully reliable [20].

### 2.5. Statistical Evaluation

The Statistical Package for Social Sciences was used to examine the data (SPSS, version 25). The chi-square test of association was used to compare proportions. Fisher's exact test was used when the expected frequency (value) was less than 5 of more than 20% of the cells of the table. A *p* value of ≤0.05 was considered statistically significant.

## 3. Results

The interexaminer reliability analysis of the readings yielded a score of 0.87, indicating that the clinical information in this study was completely accurate.

### 3.1. Prevalence of C-Shaped Canals in Mandibular Second Molars according to Age, Gender, and Tooth Position

In mandibular second molars, 64 teeth (17.4%) were found to have C-shaped canals. 47 females (23%) and 17 males (10.4%) had C-shaped canals. According to the chi-square test, the differences between males and females were very significant (*p* = 0.001). The difference between age groups and the prevalence of C-shaped canal was not significant (0.734^∗^). Furthermore, the chi-square test revealed no significant difference (0.747) between the right and left sides (Table 2).

### 3.2. Configuration of C-Shaped Canals in Mandibular Second Molars according to Age, Gender, and Tooth Position

The majority of canal orifices (36 (56.3%)) had a C2-type orifice, followed by C3 type (15 (23.4%)), C1 type, and an uninterrupted “C” shape, which had 10 (15.6%), and 3 (4.7%) of the C-shaped canals had a C4-type orifice. No statistically significant differences were found in distribution of different types of C-shaped canal configuration by age, gender, and tooth position using Fisher's exact test (Table 3, Figure 3).

### 3.3. Prevalence of C-Shaped Canals in Maxillary Second Molars according to Age, Gender, and Tooth Position

C-shaped canals were found in 29 (7.9%) of the maxillary second molars. Twenty females (9.2%) and nine males (6%) had C-shaped canals, and the differences were not significant (0.259^∗^) according to the chi-square test. Using the chi-square test, no significant relationship was detected between different age groups (0.311^∗^) and tooth position (0.201^∗^) to the prevalence of C-shaped canal (Table 4).

### 3.4. Configuration of C-Shaped Canals in Maxillary Second Molars according to Age, Gender, and Tooth Position

The most common type was type I (subtype C) (fusion of 2 root canals MB-DB) (19 (65.5%)), followed by Type I (subtype A) (fusion of 2 root canals MB-P) (6 (20.7%)). The lowest prevalence was observed for both type I (subtype B) (fusion of 2 root canals DB-P) and Type II (subtype B) (fusion of 3 root canals MB-P-DB) (1 (3.4%)). No significant differences were detected between age, gender, and tooth position with root fusions using Fisher's exact test (Table 5, Figure 4).

### 3.5. Unilateral and Bilateral Occurrence of C-Shaped Canals in Mandibular and Maxillary Second Molars to Gender

Table 5 shows the occurrence of bilateral (25 (64.1%) or unilateral (14 (35.7%) C-shaped canals in mandibular second molars, as well as bilateral (7 (46.7%) or unilateral (8 (53.3%) C-shaped canals in maxillary second molars. In mandibular second molars, most C-shaped canals were observed bilaterally in both genders, and there was no significant difference according to tooth position, while in maxillary second molars, many C-shaped canals were seen unilaterally in both genders, with no statistically significant difference regarding tooth position using Fisher's exact test (Table 6).

## 4. Discussion

The study of internal anatomy of mandibular and maxillary second molars has been the subject of numerous studies in various countries [29–31]. Second molars in the mandibular and maxillary jaws have a higher proportion of anatomical abnormalities than first molars [27, 32, 33]. The C-shaped canal has been thought to have a lot of anatomical diversity [18]. According to the literature, mandibular second molars have the largest incidence of this variation, whereas other teeth such as maxillary molars [34] and mandibular premolars [35] have also been associated to it, but with a much lower prevalence. This study is aimed at providing detailed information on C-shaped canal configuration in mandibular and maxillary second molars in an Iraqi subpopulation using CBCT.

CBCT is a nondestructive, noninvasive imaging method that can detect the majority of anatomic differences while generating an accurate description of the external and internal dental anatomy. At low radiation and dosimetry, the quality of CBCT is sufficient to visualize root canal morphology prior to endodontic therapy [36].

Differences in the occurrence of C-shaped root canal systems among races in relation to age and gender show the impact of ethnicity on the root canal morphology of mandibular and maxillary second molars. C-shaped root canals were shown to be more common in an Asian population in some research, with prevalence ranging from 2.7 percent to 8% [18, 37].  Table 7 shows the geographic location and CBCT characteristics of C-shaped canals in mandibular and maxillary second molars in each region.

Only one study [38] examined the presence of C-shaped canals in an Iraqi population, reporting an incidence of 12.1% in mandibular second molars using CBCT. In this study, CBCT was used to analyze the prevalence of C-shaped canals in both mandibular and maxillary second molars, as well as the relationship between their occurrence and age, gender, and tooth location.

Because no instances were found in the current investigation, Category V (C5) in mandibular second molars and Type II (subtype C and D) and Type III in maxillary second molars were eliminated.

In the current study, C-shaped canals were found in 17.4% of mandibular second molars. Similar percentages were reported for Venezuelan (19.5%) [31], Brazilian (15.3%) [24], and Indian (13.12%) populations [39]. However, different results were produced with Iranian (9.2%) [21], Chinese (38.6%) [26], and Korean (36.8%) [25] populations. The discrepancy could be related to differences in races, sample size, analysis technique, and statistical parameter application.

In this study, patients above the age of 50 had fewer C-shaped canals in their mandibular second molars than those under the age of 40. Patients in their 50s and 60s were also found to have fewer C-shaped canals in other studies [16, 25]. This is most likely due to secondary dentin deposition in the root canal, which can eventually obliterate the root canal space and obstruct the radiographic appearance of these anatomically complicated structures [40].

According to this study, women had a higher prevalence of C-shaped canals in their mandibular second molars than men, which was supported by some earlier studies [17, 25] but challenged by others [16, 26]. However, no variation in the prevalence of C-shaped canals in mandibular second molars was detected according to tooth location, which is consistent with the findings of other research [16, 25, 26]. It is possible that these variances are attributable to sample size and ethnic background differences. According to the findings of this study, clinicians should consider age, gender, and ethnicity when determining root canal morphology prior to root canal therapy.

Based on Fan et al.'s [18] classification, the C2 type (56.3%) was the most common type of C-shaped configurations, as reported in a study by Kim et al. [41]; however, this contradicts prior research [23, 25, 27] which indicated that both C1 and C3 types were the most prevalent at the orifice level. Differences in sample sizes and respondents' ethnic backgrounds could explain the variances. However, there was no discernible variation in the frequency of C-shaped canals in mandibular second molars based on age, gender, or tooth location.

The presence of C-shaped canals in maxillary second molars was also investigated using CBCT. A small number of studies have demonstrated the existence of C-shaped canals in maxillary second molars [19, 22, 41], because maxillary first and second molars typically have three roots with three or four root canals. Furthermore, the mandibular second molar is the most likely of the permanent teeth to exhibit this morphological variation [21, 23, 24], highlighting the importance of this study for future research.

C-shaped canals were discovered in 7.9% of maxillary second molars in this investigation. Other investigations with Colombian (12.5%) [22] and Saudi Arabian (5.1%) [42] populations yielded different results. The ethnic background, sample size, patient age, research technique, and root fusion criteria could all have a part in the disparities between studies. The prevalence of C-shaped canals in maxillary second molars was shown to be unrelated to age, gender, or tooth location. Women, on the other hand, have more C-shaped canals than men.

Our root fusion criteria for maxillary second molars were based on Ross and Evanchik's definition of a tooth having fused roots if one-third or less of the roots were fused [43]. The study indicated a decreased prevalence when an alternate criterion of considering roots fused only when fusion occurred on the complete root surface was utilized [17].

Type I, subtype C (fusion of MB and DB roots) was the most common type (65.5%) in our study, followed by Type I, subtype A (fusion of MB-P roots) and Type I, subtype B (fusion of MB and DB roots) (20.7 percent). This finding is in line with a prior Korean study [19], while a Columbian investigation found that fusion of MB and P roots was the most common kind [22]. In maxillary second molars, no significant variations were found between age, gender, tooth position, and different forms of root fusion.

In our study, the bilateral prevalence of C-shaped canals in mandibular second molars was 64.1 percent, which is comparable with studies of Korean [25] and Chinese [26] populations, but the unilateral form was more common in Brazilian [24] and Greek [28] populations. These discrepancies may be due to sample size and ethnicity. As a result, if a C-shaped canal is detected in a mandibular second molar in an Iraqi population, the contralateral second molar is likely to have one as well.

C-shaped canals were discovered unilaterally in nearly half of the maxillary second molars tested, whereas 60% of instances were identified bilaterally in a Colombian community [22].

To the authors' knowledge, this is only the second study that investigates C-shaped canals in both mandibular and maxillary second molars using CBCT in the same sample size. C-shaped canals were found in 17.4% of mandibular second molars and 7.9% of maxillary second molars in our study, according to CBCT, whereas Felsypremila et al. [44] found an overall prevalence of C-shaped canals in mandibular second molars (8.1%) and maxillary second molars (7.3%) in an Indian subpopulation (0.5%).

There are some limitations to this study; e.g., voxel size, sample size, and CBCT results came from a group of young patients (mean age: 28.33 year old for mandibular second molars and 32.86 years for maxillary second molars). As a result, extrapolating the results to the total Iraqi population based on this age distribution may be challenging.

## 5. Conclusion

In an Iraqi subpopulation, the overall prevalence of C-shaped configurations in mandibular second molars is 17.4% and that in maxillary second molars is 7.9%.

## Figures and Tables

**Figure 1:** Classification of C-shaped canal configuration in mandibular second molar by Fan et al. [18]. C1: uninterrupted C with no division or separation (a); C2: the canal shape represents a semicolon resulting from discontinuation of the C outline (b); C3: three (c) or two (d) separate canals; C4: only one round- or oval-shaped canal in the cross-section (e); C5: no canal lumen could be observed (f).

**Figure 2:** (a) Measurement of angles for the C2 canal. Angle *β* is more than 60°. (A and B) Ends of one canal cross-section; (C and D) ends of the other canal cross-section; M: middle point of line AD; *α*: angle between line AM and line BM; *β*: angle between line CM and line DM. (b) Measurement of angles for the C3 canal. Both angles *α* and *β* are less than 60°. (A and B) Ends of one canal cross-section; (C and D) ends of another canal cross-section; M: middle point of line AD; *α*: angle between line AM and line BM; *β*: angle between line CM and line DM.

**Figure 3:** Different axial portions of CBCT images of mandibular second molars with C-shaped canals: C1 (a); C2 (b, c); C3 (d, e); C4 (f). (B: buccal; L: lingual; M: mesial; D: distal).

**Figure 4:** Different axial portions of CBCT images of mandibular second molars with C-shaped canals: (a) Type I subtype A; (b) Type I subtype B; (c) Type I subtype c; (d) Type II subtype A; (e) Type II subtype B. (B: buccal; P: palatal; M: mesial; D: distal).

**Table 1:** Classification of root fusion in the maxillary second molar.

Type of root fusion		Description
Type I (fusion of 2 roots)	Subtype A (MB-P)	Mesiobuccal root fused with palatal root
	Subtype B (DB-P)	Distobuccal root fused with palatal root
	Subtype C (MB-DB)	Mesiobuccal root fused with distobuccal root
Type II (fusion of 3 roots)	Subtype A (MB-DB-P)	Mesiobuccal root fused with distobuccal root and palatal root
	Subtype B (DB-MB-P)	Distobuccal root fused with mesiobuccal root and palatal root
	Subtype C (MB-P-DB) (V shape)	Mesiobuccal root fused with palatal root and distobuccal root
	Subtype D (all roots (Y or cone shape))	All 3 roots fused to apical direction without any sequence
Type III (other types of root fusion)	Subtype A (B-P teeth with 2 roots)	Single buccal root fused with palatal root
	Subtype B (MB-MP and DB-DP)	Mesiobuccal root fused with mesiopalatal root and distobuccal root fused with distopalatal root

**Table 2:** Prevalence of C-shaped canal by age, gender, and side in mandibular second molars.

	Prevalence of C shape						
	Present		Absent		Total		
	No.	(%)	No.	(%)	No.	(%)	*p*
Age (years)							
<30	40	(17.5)	189	(82.5)	229	(100.0)	
30-39	22	(19.1)	93	(80.9)	115	(100.0)	
40-49	2	(11.8)	15	(88.2)	17	(100.0)	
≥50	0	(0.0)	7	(100.0)	7	(100.0)	0.734^∗^
Gender							
Male	17	(10.4)	147	(89.6)	164	(100.0)	
Female	47	(23)	157	(77.0)	204	(100.0)	0.001^†^
Side							
Right	31	(16.8)	154	(83.2)	185	(100.0)	
Left	33	(18.0)	150	(82.0)	183	(100.0)	0.747^†^
Total	64	(17.4)	304	(82.6)	368	(100.0)	

^∗^By Fisher's exact test. ^†^By the chi-square test.

**Table 3:** Classification of C-shaped canal by age, gender, and side in the mandibular second molars.

	Categories of C-shaped canal^†^				
	C1	C2	C3	C4	
	No. (%)	No. (%)	No. (%)	No. (%)	*p*
Age (years)					
<30	6 (15.0)	19 (47.5)	12 (30.0)	3 (7.5)	
30-39	3 (13.6)	17 (77.3)	2 (9.1)	0 (0.0)	
40-49	1 (50.0)	0 (0.0)	1 (50.0)	0 (0.0)	0.060^∗^
Gender					
Male	3 (17.6)	8 (47.1)	6 (35.3)	0 (0.0)	
Female	7 (14.9)	28 (59.6)	9 (19.1)	3 (6.4)	0.505^∗^
Side					
Right	4 (12.9)	18 (58.1)	8 (25.8)	1 (3.2)	
Left	6 (18.2)	18 (54.5)	7 (21.2)	2 (6.1)	0.928^∗^
Total	10 (15.6)	36 (56.3)	15 (23.4)	3 (4.7)	

^∗^By Fisher's exact test. C1: uninterrupted “C” with no separation or division. C2: a semicolon resulting from a discontinuation of the “C” outline, but either the *α* or *β* angle should be no less than 60°. C3: two or 3 separate canals and both angles, *α* and *β*, were less than 60°. C4: a single round or oval canal.

**Table 4:** Prevalence of C-shaped canal by age, gender, and side in maxillary second molars.

	Prevalence of C-shape						
	Present		Absent		Total		
	No.	(%)	No.	(%)	No.	(%)	*p*
Age (years)							
<30	16	(10.9)	131	(89.1)	147	(100.0)	
30-39	8	(6.2)	122	(93.8)	130	(100.0)	
40-49	3	(4.3)	66	(95.7)	69	(100.0)	
≥50	2	(8.7)	21	(91.3)	23	(100.0)	0.311^∗^
Gender							
Male	9	(6.0)	142	(94.0)	151	(100.0)	
Female	20	(9.2)	198	(90.8)	218	(100.0)	0.259^∗^
Side							
Right	18	(9.6)	169	(90.4)	187	(100.0)	
Left	11	(6.0)	171	(94.0)	182	(100.0)	0.201^∗^
Total	29	(7.9)	340	(92.1)	369	(100.0)	

^∗^By the chi-square test.

**Table 5:** Classification of C-shaped canal by age, gender, and side in maxillary second molars.

	Categories of C-shaped canal^†^					
	Type I (subtype A)	Type I (subtype B)	Type I (subtype C)	Type II (subtype A)	Type II (subtype B)	
	No. (%)	No. (%)	No. (%)	No. (%)	No. (%)	*p*
Age (years)						
<30	2 (12.5)	0 (0.0)	12 (75.0)	1 (6.3)	1 (6.3)	
30-39	3 (37.5)	0 (0.0)	4 (50.0)	1 (12.5)	0 (0.0)	
40-49	1 (33.3)	1 (33.3)	1 (33.3)	0 (0.0)	0 (0.0)	
≥50	0 (0.0)	0 (0.0)	2 (100.0)	0 (0.0)	0 (0.0)	0.391^∗^
Gender						
Male	3 (33.3)	0 (0.0)	5 (55.6)	0 (0.0)	1 (11.1)	
Female	3 (15.0)	1 (5.0)	14 (70.0)	2 (10.0)	0 (0.0)	0.361^∗^
Side						
Right	5 (27.8)	0 (0.0)	11 (61.1)	2 (11.1)	0 (0.0)	
Left	1 (9.1)	1 (9.1)	8 (72.7)	0 (0.0)	1 (9.1)	0.211^∗^
Total	6 (20.7)	1 (3.4)	19 (65.5)	2 (6.9)	1 (3.4)	

^∗^By Fisher's exact test. Type I (subtype A): Type I fusion of 2 root canals-subtypes A (MB-P). Type I (subtype B): Type I fusion of 2 root canals-subtypes B (DB-P). Type I (subtype C): Type I (fusion of 2 root canals)-subtype C (MB-DB). Type II (subtype A): Type II fusion of 3 root canals-subtypes A DB-MB-P. Type II (Subtype B): Type II fusion of 3 root canals-subtypes B (MB-P-DB) (V shape).

**Table 6:** Occurrence of bilateral/unilateral C-shaped canal in mandibular and maxillary second molars by gender.

	Prevalence of bilateral C-shaped canal						
	Unilateral		Bilateral		Total		
	No.	(%)	No.	(%)	No.	(%)	*p*
*Mandibular second molar*							
Gender							
Male	4	(44.4)	5	(55.6)	9	(100.0)	
Female	10	(33.3)	20	(66.7)	30	(100.0)	0.696^∗^
Total	14	(35.9)	25	(64.1)	39	(100.0)	
*Maxillary second molar*							
Gender							
Male	2	(50.0)	2	(50.0)	4	(100.0)	
Female	6	(54.5)	5	(45.5)	11	(100.0)	0.999^∗^
Total	8	(53.3)	7	(46.7)	15	(100.0)	

^∗^By Fisher's exact test.

**Table 7:** C-shaped canal configurations found in mandibular and maxillary second molars in previous studies assessed by CBCT.

References	Region/race	Teeth studied	Number of teeth	Prevalence of C-shaped canal	Classification	Unilateral/bilateral occurrence
Donyavi et al. [21]	Iran	Mandibular second molars	447	9.2%	—	—
Marcano-Caldera et al. [22]	Colombia	Maxillary second molars	740	12.5%	-Type II, subtype D (45.3%) -Type I, subtype A (MB-P) (21.5%)	—
Jo et al. [19]	Korea	Maxillary second molars	1767	2.7%	-Type I, subtype C (MB-DB) (1.6%) -Type I, subtype A (MB-P) (0.6%)	—
Mashyakhy et al. [23]	Saudi	Mandibular second molars	367	7.9%	-C3 (35.6%) -C1 (23.0%) -C2 (20.7%) -C4 (18.4%)	-Right side absence (96.4%) present (3.6%) -Left side absence (94.8%) present (5.2%)
Ladeira et al. [24]	Brazil	Mandibular second molars	406	15.3%	-Three canals (43.5%) -Two canals (37.1%)	-Unilateral C-shaped (68.3%)
Yang et al. [25]	Korea	Mandibular second molars	2508	36.8%	-C1 (35.3%) -C3b (21.6%) -C2 (21.2%) -C3a (17.5%) -C4 (4.4%)	-Bilateral C-shaped (85.9%)
Zheng et al. [26]	China	Mandibular second molars	688	38.6%	-C1 (72.5%) -C2 (18.1%) -C3 (7.8%)	-Bilateral C-shaped (81%) -Left side (12.5%) -Right side (6.3%)
Martins et al. [27]	Portugal	Mandibular second molars	1088	8.5%	-C3 (38.1%) -C2 (23.4%) -C1 (21.1%) -C4 (17.2%)	-Left side (7.6%) -Right side (9.5%)
Kantilieraki et al. [28]	Greek	Mandibular second molars	524	10.8%	-C1 (77.4%) -C3b (15.1%) -C3a (7.5%)	-Unilateral C-shaped (75.5%) -Bilateral C-shaped (24.5%)
Present study	Iraq	Mandibular second molars	368	17.4%	-C2 (56.3%) -C3 (23.4%) -C1 (15.6%) -C4 (4.7%)	-Unilateral C-shaped (35.9%) -Bilateral C-shaped (64.1%)
		Maxillary second molars	369	7.9%	-Type I, subtype C (MB-DB) (65.5%) -Type I, subtype A (MB-P) (20.7%) -Type II, subtype A (DB-MB-P) (20.7%) -Type I, subtype B (DB-P) (3.4%) -Type II, subtype B (MB-P-DB) (3.4%)	-Unilateral C-shaped (53.3%) -Bilateral C-shaped (46.7%)

CBCT: cone-beam computed tomography; DB: distobuccal; MB: mesiobuccal; P: palatal.

## Data Availability

The data used to support the findings of this study are available from the corresponding author upon reasonable request.
